# Association of Training in Basic Life Support with the Evolution of Cardiopulmonary Resuscitation Performed by Firefighters

**DOI:** 10.1155/2023/8150697

**Published:** 2023-05-05

**Authors:** Marcelo Donizeti Silva, Ricardo Augusto Barbieri, Yan Figueiredo Foresti, Jônatas Augusto Cursiol, Fernando Antônio Viana, Ednei Fernando dos Santos, Karine Pereira Rodrigues, Guilherme da Silva Rodrigues, Juliana da Silva Garcia Nascimento, Maria Celia Barcellos Dalri

**Affiliations:** ^1^School of Nursing of Ribeirao Preto, University of Sao Paulo, Avenida Bandeirantes 3900, 14049-900 Ribeirao Preto, São Paulo, Brazil; ^2^School of Physical Education and Sport of Ribeirao Preto, University of Sao Paulo, Avenida Bandeirantes 3900, 14049-900 Ribeirao Preto, São Paulo, Brazil; ^3^Sports School of the Military Police of São Paulo State, São Paulo, Brazil; ^4^Department of Internal Medicine, Ribeirão Preto Medical School, University of São Paulo, São Paulo, Brazil

## Abstract

**Introduction:**

This study aimed to compare the results of professional technical and anthropometric anamnesis data with the transmission of external chest compressions performed by military firefighters at different execution times.

**Objective:**

The objective was to evaluate the performance and perceived effort of the sequence of external chest compressions performed in two minutes, as well as the evolution of the technique over time.

**Materials and Methods:**

This was a descriptive, correlational study involving adult firefighters who were members of a specific firefighter group, comprising a population of 105 individuals with a voluntary sample of 44 participants. The study used a Bayesian statistical approach to provide probabilistic expressions.

**Results:**

The participants had an average work experience of 17 years, an average age of 38.6 years, an average weight of 81.48 kilograms, an average height of 176 centimeters, and an average of 2.5 qualifications. The results indicated that the firefighters performed external chest compressions with excellent technique and a moderate level of perceived effort in a two-minute evaluation. The evaluation of the evolution of the technique over time showed that the participants were able to maintain high-quality compressions for an average of 6 minutes, with a maximum of 20 uninterrupted minutes.

**Conclusion:**

The study underscores the critical role of professional firefighters in performing and maintaining high-quality external chest compressions, which has the potential to reduce morbidity and mortality in cases of cardiorespiratory arrest.

## 1. Introduction

The performance of cardiopulmonary resuscitation (CPR) in pre-hospital care settings is crucial, particularly when carried out by well-trained teams in large networks. In Brazil, the Fire Department plays a vital role in these situations as they frequently respond to out-of-hospital cardiorespiratory arrests (CRA) and perform CPR using motorcycles and rescue vehicles. CPR is the primary intervention for CRA, as it helps to maintain blood circulation, and its prompt implementation is one of the key factors in the success of resuscitation for individuals who experience CRA outside of a hospital setting, thereby significantly increasing their chances of survival [1–5]. Effective CPR requires external chest compressions (ETCs) at a rate of 100 to 120 movements per minute and a depth of 5 to 6 centimeters in adults, emphasizing the importance of good-quality CPR and its timely implementation [1]. However, performing high-quality CPR can lead to rescuer fatigue [6, 7] causing a decrease in the quality of ETCs during CPR after two minutes [8, 9], which is why it is recommended that rescuers be replaced every two minutes [1].

The Ministry of Health's Ordinance 2048 (2002) establishes and regulates Pre-Hospital Care (APH) services in Brazil. In the State of São Paulo, the Fire Department, as part of the Military Police, is responsible for pre-hospital APH care. Their goal is to provide prompt and appropriate care, stabilize the patient's vital signs, reduce morbidity and mortality, and quickly transport the patient to adequate medical care.

To achieve these goals, it is essential to work in large networks and with well-trained teams. In Brazil, the Fire Department plays a crucial role in these services, providing daily support to health units with motorcycles and rescue vehicles. They are usually the first professionals to face out-of-hospital CPA and are capable of performing cardiopulmonary resuscitation (CPR).

In the ambulance, the rescue team of the Fire Department comprises three rescuers who provide hands-on assistance in any occurrence. They are not authorized to administer medication or perform invasive procedures. The Fire Department's response time, from receiving the call to the arrival of the vehicles to attend to the occurrence, is approximately 10 minutes in Brazil.

Basic Life Support (BLS) training is critical for providing care to patients in CRA in out-of-hospital environments [1], but even with training, people still sometimes fail to perform chest compressions during [10]. Hence, the ongoing training of rescuers is crucial for providing life support in cardiovascular emergencies [11–13]. The monitoring of ETCs during training and further scientific research into the effectiveness of these procedures is a critical need in the field of CPR [14]. The present study aimed to investigate the relationship between BLS training and the effectiveness of CPR performed by firefighters and to examine the association between the amount of training received and the time of voluntary interruption due to rescuer fatigue during the performance of ETCs. The hypothesis of the study was that firefighters with more BLS training would exhibit higher effectiveness in CPR, with a focus on ETCs, and would have a longer duration of effective CPR performance before voluntarily interrupting due to exhaustion.

## 2. Materials and Methods

The target population of this study was adult firefighters working at the 9th Group of Firefighters in the city of Ribeirão Preto, São Paulo. The sample was voluntary and consisted of 105 firefighters, but only 44 of them who fully participated in all stages of the study were included. The inclusion criteria were being a firefighter working in Ribeirão Preto and exclusion criteria was being on sick leave, leave, or vacation during the data collection period. The sample size was calculated using *G* ^*∗*^ Power software (version 3.1, University of Düsseldorf) based on a predicted effect size of 0.4 and a desired power of 80% at an alpha level of 0.05 [15]. The study was approved by the Ethics and Research Committee and registered at Plataforma Brasil with CAAE 10431719.9.0000.5393. The data collection took place from January to November 2020, including the interruption of activities due to the Covid-19 pandemic.

This study is a descriptive and correlational investigation comparing the results of professional technical anamnesis with the performance of CPR, with a focus on chest compressions, among military firefighters. The study was conducted in four stages at the Command Headquarters of the 9th Group of Firefighters in Ribeirão Preto, São Paulo. The execution time of CPR was two minutes or until voluntary exhaustion (Figure 1).

  The first stage—invitation and participants characterization: Participants were contacted personally in the five barracks of the 9th Group of Firefighters located in Ribeirão Preto, São Paulo. The study was introduced to the participants, and those who consented signed an Informed Consent Form (ICF) and completed the technical-professional anamnesis form. The technical-professional anamnesis was conducted through a questionnaire designed by the researchers as a control mechanism and for characterizing the participants. The data collected from the questionnaire and throughout the study were only used for the purposes explicitly stated in the ICF. The questionnaire was developed by the researcher and included information such as the participant's name, gender, date of birth, marital status, academic background, date of admission to the corporation, firefighter specialization courses, and physical activity practices.
  The second stage—theoretical-practical training: The volunteers underwent theoretical and practical training, which lasted approximately 15 minutes in the theoretical component. During this time, they received an update on CPR/CPR and CTEs in accordance with the guidelines recommended by the American Heart Association [1] for Basic Life Support (BLS). Then, they underwent two practical CPR training sessions, with an emphasis on CTEs, using a Laerdal Resusci Anne Wireless SkillReporter manikin. This manikin provides real-time feedback to the participant during the training, allowing for high-performance practical skills training for healthcare professionals and first responders. The manikin offers precise and proficient CPR training, enabling the use of protocols, equipment, and techniques used in real-life situations. To ensure standardization and proximity to real-life scenarios, the participants were dressed in the operational work clothes of firefighters and wore gloves for procedures and a surgical mask. At the end of the CPR simulations, a feedback report was generated by the manikin and entered into a Microsoft Excel database for statistical analysis. In the first period of practical training, participants performed two minutes of CTEs with feedback, along with verbal encouragement from the evaluators. In the second training period, after approximately 30 minutes of rest, the volunteers performed the CTEs again, until they voluntarily stopped due to exhaustion, with feedback on the effectiveness of the CTEs (frequency and depth) and verbal encouragement from the evaluators.
  The third stage—evaluation of the effectiveness of CPR with a focus on chest compression techniques: After a minimum interval of 48 hours and a maximum of one week, the volunteers performed chest compression techniques on the Laerdal Resusci Anne Wireless SkillReporter manikin, lasting for two minutes, without receiving feedback from the manikin or evaluators. In this stage, the effectiveness of the chest compressions performed by the participants was assessed. The participants' initial and final heart rates were recorded before and after each test, respectively.
  The fourth stage—CTE effectiveness test with emphasis on CTEs: After a minimum period of 48 hours and a maximum of one week, participants performed CTEs on a manikin, continuing until voluntary exhaustion, with no feedback from either the manikin or evaluators. At this stage, the effectiveness of the CTEs performed by the participants until voluntary exhaustion was evaluated. The participant's initial and final heart rate was checked at the beginning and end of each test. Statistical analyses were performed using JASP software (Amsterdam, Netherlands) version 0.12.2. A Bayesian statistical approach was employed to provide probabilistic assertions, as it offers a valuable alternative to interpreting the relative support of a null hypothesis against an alternative hypothesis [16, 17]. The normality of data distribution was confirmed using *Q-Q* plots, and data are reported as mean ± standard deviation (SD). The Bayes Factor (BF10) was calculated for all variables using the “uninformative” hypothesis predefined by JASP (Cauchy, 0.707). Evidence for the alternative hypothesis (H1) was established as BF10 > 3 and evidence for the null hypothesis (H0) as BF10 < 1/3. BF calculates the probability that the null (H0) or alternative (H1) hypothesis is true given the current data. In case of a significant H1-favorable Bayes Factor (BF10), a post hoc analysis was performed [18]. BF10 was reported to indicate the strength of evidence for each analysis (within and between) and interpreted as anecdotal (BF10 = 1–3), moderate (BF10 = 3–10), strong (BF10 = 10–30), very strong (BF10 = 30–100) when favoring the alternative hypothesis; or anecdotal (BF10 = 1–0.33), moderate (BF10 = 0.33–0.01), strong (BF10 = 0.01–0.03), very strong (BF10 = 0.03–0.01), and extreme (BF10 < 0.01) when favoring the null hypothesis [19].

## 3. Results

In Table 1, the characterization of the participants is presented regarding the variables obtained in the technical-professional anamnesis. Of the 44 (100%) professional firefighters who made up the sample in this study, all were male. The mean of the subjective scale of perceived exertion (3.00), during the CTEs, was considered moderate (Table 2).

Table 3, presents the correlation between the variables referring to the characterization of the professional firefighter and the effectiveness of the CTEs in the two-minute test. The analysis regarding the relationship between the presence of training/specialization courses for firefighters and the effectiveness of CTEs performed within two minutes showed that there is a moderate correlation between the number of courses taken and the reduction of subjective fatigue during the two-minute effort. Specifically, the more training sessions taken, the greater the positive impact on reducing the feeling of fatigue during CTEs.

Table 4 presents the results of the assessment of the effectiveness of CPR via the voluntary interruption test (time to exhaustion). The assessment of the effectiveness of the CTEs based on the time to exhaustion revealed that, primarily, the maximum time that participants were able to perform CTEs with quality and effectiveness was 20 uninterrupted minutes. Only one participant was unable to reach the minimum required time of two minutes. Although the participants rated the difficulty level during the evaluation as 4.80, it was considered relatively manageable. The correlation between the characteristics of professional firefighters and the effectiveness of the CTEs as determined by the time to exhaustion test is presented in Table 5.

The analysis of the relationship between the effectiveness of CTEs until exhaustion and variables pertaining to the characterization of participants in the present study revealed a moderate negative correlation between the body weight of the firefighters and the ability to maintain proper hand placement on the victim's chest during compressions. In other words, a greater body weight among professionals was associated with increased difficulty in maintaining proper hand placement during the CTEs.

## 4. Discussion

The objective of this study was to examine the relationship between basic life support training and the effectiveness of cardiopulmonary resuscitation (CPR) performed by firefighters and to assess the correlation between the amount of training received and the time of voluntary interruption due to exhaustion during CPR. Despite the significance of CPR in an out-of-hospital environment and the crucial role played by firefighters in performing CPR [20], studies on the relationship between physical fitness, body composition, and the effectiveness of CPR typically do not consider firefighters as a distinct population [21], highlighting the need and importance of addressing this demographic in this context [9, 12].

In line with this objective, this study recruited 44 male professional firefighters as participants. Most of them were experienced in their field, adults, and had an average body weight and height that is typical for their profession [22, 23]. Other studies that have studied firefighters as a population have similar sample characteristics and inclusion criteria as this research [22, 24–26].

The average number of training courses and specializations taken by the participants was 2.5, with 10 professionals having not taken any specialization courses. The teaching and learning processes adopted for firefighter training are of interest to the fields of health, education, and resuscitation, as developing these skills is essential for the profession [27]. A moderate correlation was found in the study between the number of courses taken and the decrease in feelings of subjective fatigue during two-minute CPR efforts. This indicates that greater technical-scientific preparation results in less difficulty and fatigue perceived during CPR.

Ferreira Junior et al. found a correlation between CPR knowledge and age among firefighters, with those under 35 having gaps in CPR knowledge due to a lack of specialized training and a lack of variety of training necessary for developing knowledge, skills, and attitudes for daily practice [28]. This can negatively impact the quality of CPR and increase fatigue during the procedure. Adopting simulator mannequins is becoming increasingly popular for firefighter training as they enable the development of psychomotor skills necessary for professional practice [27].

Regardless of the number of events in which a soldier has participated throughout his career, no two situations will ever be identical. The variables involved, such as the characters, psychological and material conditions, external interferences, and risks to be overcome, all differ. To address this variability of events, technical-scientific preparation is necessary, which can be enhanced through courses and training conducted during professional experience [29].

The effectiveness of cardiopulmonary resuscitation (CPR) procedures (CTEs) was found to be of interest, a priori, in a time frame of two minutes. Firefighters were observed to perform the procedure well within this time frame, with an average perceived exertion score classified as moderate. However, this finding can negatively impact the quality of the CTE and increase fatigue during the procedure [28]. In another perspective, a cross-sectional study with 63 university students trained in CPR analyzed the relationship between muscle strength and CTEs and concluded that the ability to provide effective CTEs is influenced by the rescuer's muscle strength, with individuals of lower weight having lower results, particularly in terms of correct compression depth, compared to those with normal weight and those with overweight/obesity [30].

A similar cross-sectional study of 48 trained rescuers, aged between 26 and 46 years, aimed to perform CTEs on a simulator dummy until they reached the maximum reported level of fatigue. The average duration of the CTEs was 3.28 minutes with a standard deviation of 1.04 minutes, with better times being achieved by those with higher levels of physical activity. This study concluded that the greater the physical preparation, the lower the level of fatigue and the greater the duration of the CTEs [9]. Maintaining a CTE time of approximately 5 minutes and reaching 20 uninterrupted minutes with a level of fatigue classified as “a little difficult” are important findings of the present study, as the literature typically describes rescuer fatigue within the first minute of CTE [9, 31, 32]. It is possible that a rescuer who is capable of performing a high-quality CTE for a longer duration has a high level of physical training, which positively impacts the reduction of fatigue and maintains their muscular, physical, and cardiorespiratory capacity, ensuring their ability to effectively perform the CTE [33].

The Voluntary Interruption Test revealed that a professional's body weight affects their ability to maintain hand contact with the thoracic region during compressions. A cross-sectional study involving 63 university students previously trained in CPR found that the rescuer's muscle strength impacts their ability to perform effective compressions. This study concluded that individuals with low weight had lower results in terms of compression depth, compared to those with normal weight and those with overweight/obesity [31]. This suggests that variations in weight, whether low or high, can negatively impact the quality of compressions. Further studies are necessary to confirm these findings [34, 35].

The limitations of this work included the scarcity of literature regarding the relationships between physical fitness, body composition, and the effectiveness of compressions, particularly among professional firefighters. This makes it challenging to compare results in different scenarios. Nevertheless, this did not hinder the analysis and interpretation of the results.

More research is needed in this area, specifically well-designed studies with a high level of evidence, to evaluate the effectiveness of compressions in different groups of rescuers with varying body compositions. This will contribute greatly to research, teaching, and assistance.

## 5. Conclusion

Specifically, the evaluation of CTE effectiveness, conducted over two minutes, indicated excellent performance by firefighters and a moderate level of perceived effort during compressions. The voluntary interruption test for exhaustion showed that, on average, the participants were able to perform high-quality compressions for up to 6 minutes, with some reaching as much as 20 uninterrupted minutes. The subjective perception of fatigue during this test was described as manageable.

This study is significant because of the crucial role professional firefighters play in performing effective CTEs, which can impact the reduction of morbidity and mortality in CPR cases. The results of this research have multiple implications, including the development of training and educational strategies tailored to professional firefighters, improvement in the quality of CTEs performed by firefighters, and the potential to replicate these findings in other professional fields to promote education, research, and assistance in CPR. This knowledge can also contribute to the improvement of patient safety and quality of care in CPR, particularly in terms of high-quality compressions. This study highlights the importance of a multidisciplinary approach to care, encompassing fields such as nursing, firefighting, and physical education, in the pursuit of life-saving knowledge.

## Figures and Tables

**Figure 1:** Research flowchart. Source: by the author, 2022.

**Table 1:** Characterization of firefighters regarding the variables obtained in the technical-professional anamnesis.

Variable	Average	SD	Minimum	Maximum
Age (years)	38.68	5.44	27	52
Weight (kg)	81.48	10.95	55	112
Height (cm)	176.09	5.52	165	189
Admission to the corporation (months)	205.48	82.34	58	376
Training/specialization courses (*n*)	2.25	2.06	0	7

kg: kilogram; cm: centimeters.

**Table 2:** Distribution of firefighters according to the variables of effectiveness of external chest compressions performed on a dummy, the subjective perception of effort and the heart rate of the participants, in two minutes.

Variable	Average	SD	Minimum	Maximum
Total performance (%)	96.98	4.08	81	100
Quality of CTEs (%)	97.25	3.65	81	100
Contact of hands-on chest (%)	99.77	1.22	92	100
Test time (min)	2.0	0.0	2	2
Absence of CTEs (sec)	0.11	0.39	0	2
Correct hand position (%)	98.68	4.01	82	100
Total number of compressions	221.68	15.08	183	259
Mean depth (mm)	55.77	3.45	50	61
Adequate chest return (%)	89.75	19.68	0	100
Compression force (%)	93.55	12.15	56	100
Adequate pace of CTEs (%)	85.09	26.18	0	100
Average CTEs per minute	110.48	7.1	92	129

*Firefighter*				
Heart rate start	77.93	11.81	52	101
Final heart rate	99.68	17.59	66	150
PSE scale	3.0	0.96	1	5

PSE scale: perceived exertion scale; sec: seconds; min: minutes. *Note*. Data are expressed as mean and standard deviation, in addition to the minimum and maximum parameters.

**Table 3:** Correlation between firefighter characterization variables and the effectiveness of external chest compressions in two minutes.

Teste CTEs 2 min	Service time		Training/specialization courses		Age		Weight		Stature	
	Pearson's *r*	BF₁₀	Pearson's *r*	BF₁₀	Pearson's *r*	BF₁₀	Pearson's *r*	BF₁₀	Pearson's *r*	BF₁₀
Total performance (%)	0.171	0.342	0.217	0.494	0.024	0.19	−0.178	0.36	0.025	0.19
Quality of CTEs (%)	0.175	0.35	0.23	0.557	0.008	0.188	−0.108	0.238	−0.044	0.195
Contact of hands-on chest (%)	0.044	0.195	0.032	0.192	0.052	0.198	−0.21	0.464	0.18	0.363
Absence of CTEs (sec)	0.004	0.188	−0.066	0.205	−0.17	0.34	−0.068	0.206	−0.255	0.728
Correct hand position (%)	−0.011	0.188	−0.092	0.222	−0.068	0.206	−0.113	0.243	−0.04	0.194
Total number of compressions	−0.006	0.188	0.115	0.245	0.095	0.226	0.016	0.189	0.156	0.307
Mean depth (mm)	0.086	0.218	−0.008	0.188	0.167	0.332	0.247	0.669	−0.01	0.188
Adequate chest return (%)	0.193	0.403	0.171	0.341	0.179	0.361	−0.039	0.194	0.041	0.194
Compression force (%)	0.123	0.255	0.089	0.221	0.027	0.191	0.095	0.225	0.074	0.21
Adequate pace of CTEs (%)	0.033	0.192	0.136	0.274	0.027	0.191	−0.166	0.329	−0.116	0.247
Average CTEs per minute	−0.014	0.189	0.113	0.243	0.1	0.23	0.05	0.197	0.066	0.205

*Firefighter*										
Heart rate start	−0.155	0.307	−0.131	0.266	−0.158	0.311	0.035	0.193	0.101	0.231
Final heart rate	−0.098	0.228	−0.127	0.26	−0.232	0.57	−0.053	0.199	0.047	0.196
PSE scale	−0.238	0.605	**−0.375**	^*∗*^ ** 3.932**	0.275	0.911	0.064	0.204	−0.004	0.188

PSE scale = perceived exertion scale. Bold results indicate significant correlations at *p* > 0.05. *Note.* “*r*” corresponds to Pearson's Bayesian correlation and “BF₁₀” corresponds to the Bayes factor, where ^*∗*^BF₁₀ between 3 and 10 (moderate); ^*∗∗*^BF₁₀ between 10 and 30 (strong); ^*∗∗∗*^BF₁₀ between 30 and 100 (very strong); ^*∗∗∗∗*^BF₁₀ > 100 (extreme).

**Table 4:** Distribution of firefighters according to the variables of effectiveness of external chest compressions performed on a dummy, the subjective perception of effort and the heart rate of the participants, until the time of exhaustion.

Variable	Average	SD	Minimum	Maximum
Total performance (%)	96.11	5.72	65	100
Quality of CTEs (%)	96.48	5.63	66	100
Contact of hands-on chest (%)	99.36	0.92	96	100
Test time (min)	5.64	4.94	1.43	20
Absence of CTEs (sec)	1.23	1.49	0	4
Correct hand position (%)	98.55	4.52	78	100
Total number of compressions	641.41	534.74	215	2379
Mean depth (mm)	55.82	4.05	49	67
Adequate chest return (%)	91.59	17.18	22	100
Compression force (%)	92.55	14.08	38	100
Adequate pace of CTEs (%)	83.09	28.28	0	100
Average CTEs per minute	112.09	7.69	93	140

*Firefighter*				
Heart rate start	79.82	11.24	53	103
Final heart rate	108.46	17.07	68	154
PSE scale	4.8	1.52	2	9

PSE scale: perceived exertion scale; min: minutes. *Note*. Data are expressed as mean and standard deviation, in addition to the minimum and maximum parameters.

**Table 5:** Correlation between the firefighter characterization variables and the effectiveness of external chest compressions, up to the time of exhaustion.

Testing of CTEs in exhaustion time	Service time		Training/specialization courses		Age		Weight		Stature	
	Pearson's *r*	BF₁₀	Pearson's *r*	BF₁₀	Pearson's *r*	BF₁₀	Pearson's *r*	BF₁₀	Pearson's *r*	BF₁₀
Total performance (%)	−0.183	0.372	0.248	0.675	−0.272	0.878	−0.125	0.258	0.111	0.241
Quality of CTEs (%)	−0.176	0.353	0.248	0.676	−0.272	0.876	−0.086	0.218	0.124	0.256
Contact of hands-on chest (%)	−0.224	0.527	0.049	0.197	−0.149	0.295	**−0.365**	^*∗*^ ** 3.327**	−0.066	0.205
Test time (min)	0.092	0.223	0.129	0.263	−0.054	0.199	0.229	0.553	0.15	0.297
Absence of CTEs (sec)	0.169	0.335	−0.026	0.191	0.049	0.197	0.299	1.239	0.201	0.429
Correct hand position (%)	−0.05	0.197	−0.022	0.19	−0.099	0.229	−0.014	0.189	0.094	0.224
Total number of compressions	0.088	0.22	0.098	0.228	−0.074	0.21	0.213	0.477	0.157	0.311
Mean depth (mm)	0.205	0.446	0.307	1.365	−0.11	0.24	−0.029	0.191	−0.15	0.297
Adequate chest return (%)	−0.346	2.443	−0.097	0.227	0.156	0.309	−0.295	1.177	−0.121	0.253
Compression force (%)	0.092	0.223	0.292	1.128	0.083	0.216	0.068	0.206	−0.166	0.33
Adequate pace of CTEs (%)	−0.172	0.342	0.133	0.268	−0.291	1.109	−0.251	0.696	0.137	0.275
Average CTEs per minute	0.036	0.193	−0.289	1.087	−0.092	0.223	0.067	0.206	0.057	0.201

*Firefighter*										
Heart rate start	−0.174	0.348	−0.205	0.445	−0.127	0.26	−0.046	0.196	−0.012	0.188
Final heart rate	−0.055	0.2	−0.046	0.196	−0.209	0.461	0.192	0.401	0.021	0.19
PSE scale	−0.088	0.22	−0.154	0.305	0.023	0.19	0.203	0.439	−0.062	0.203

PSE scale: perceived exertion scale; sec: seconds. Bold results indicate significant correlations at *p* > 0.05. *Note.* “*r*” corresponds to Pearson's Bayesian correlation and “BF₁₀” corresponds to the Bayes factor, where ^*∗*^BF₁₀ between 3 and 10 (moderate); ^*∗∗*^BF₁₀ between 10 and 30 (strong); ^*∗∗∗*^BF₁₀ between 30 and 100 (very strong); ^*∗∗∗∗*^BF₁₀ > 100 (extreme).

## Data Availability

Readers can access the data through the tables and figures available in the manuscript, and if they want to check in depth, they should contact the authors by e-mail.
